# Gambogenic acid alters chemosensitivity of breast cancer cells to Adriamycin

**DOI:** 10.1186/s12906-015-0710-8

**Published:** 2015-06-12

**Authors:** Ye He, Jie Ding, Yan Lin, Juan Li, Yongguo Shi, Juan Wang, Ya Zhu, Keming Wang, Xuezhen Hu

**Affiliations:** Department of Oncology, Wuhu NO.2 People’s Hospital, Wuhu, Anhui PR China; Department of Oncology, Second Affiliated Hospital, Nanjing Medical University, Nanjing, Jiangsu PR China; Jiangsu Province Hospital of TCM, Affiliated Hospital of Nanjing University of TCM, Nanjing, Jiangsu PR China

**Keywords:** Gambogenic acid, Breast cancer, Akt

## Abstract

**Background:**

Breast cancer remains a major health problem worldwide, and is becoming increasingly resistant to traditional drug treatments. For instance, Adriamycin (ADR) is beneficial for the treatment of breast cancer. However, its wide application often leads to drug resistance in clinic practice, which results in treatment failure. Gambogenic acid (GNA), a polyprenylated xanthone isolated from the traditional medicine gamboge, has been reported to effectively inhibit the survival and proliferation of cancer cells. Its effects on ADR resistance have not yet been reported in breast cancer. In this study, we examined the ability of GNA to modulate ADR resiatance and the molecular mechanisms underlying this process using a cell based in vitro system.

**Methods:**

An MTT assay was used to evaluate the inhibitory effect of the drugs on the growth of MCF-7 and MCF-7/ADR cell lines. The effects of drugs on apoptosis were detected using Annexin-V APC/7-AAD double staining. The expression of apoptosis-related proteins and the proteins in the PTEN/PI3K/AKT pathway were evaluated by Western blot analysis.

**Results:**

In the MCF-7/ADR cell lines, the IC50 (half maximal inhibitory concentration) of the group that received combined treatment with GNA and ADR was significantly lower than that in the ADR group, and this value decreased with an increasing concentration of GNA. In parallel, GNA treatment increased the chemosensitivity of breast cancer cells to ADR. The cell apoptosis and cell cycle anaysis indicated that the anti-proliferative effect of GNA is in virtue of increased G0/G1 arrest and potentiated apoptosis. When combined with GNA in MCF-7/ADR cell lines, the expression levels of the tumor suppressor gene PTEN (phosphatase and tensin homolog deleted on chromosome ten) and the apoptosis-related proteins caspase-3 and capsese-9 were significantly increased, while the expression of phosphorylated AKT was decreased.

**Conclusions:**

Our study has indicated a potential role for GNA to increase the chemosensitivity of breast cancer cells to ADR. This modulatory role was mediated by suppression of the PTEN/PI3K/AKT pathway that led to apoptosis in MCF-7/ADR cells. This work suggests that GNA may be used as a regulatory agent for treating ADR resistance in breast cancer patients.

## Background

Breast cancer is one of the most common types of malignancy in Western countries [1], and its incidence is increasing in Asian countries, such as China [2, 3]. Despite the improved prognosis of breast cancer patients because of early diagnosis, radical surgery and the development of adjuvant therapy, this disease still remains a major health problem worldwide. Breast cancer is found mainly in premenopausal women older than 35 years. The incidence is associated with people’s living habits,biological factors, social factors, etc. [4]. Currently, chemotherapy is one of the most important approaches in the treatment of breast cancer [5–7]. Adriamycin (ADR) has been one of the most effective anti-cancer agents to treat solid tumors [8], including breast cancer, since its inception [9]; however, the wide application of ADR has often led to drug insensitivity, drug resistance and other phenomena in the clinic, leading to treatment failure. Thus, finding a novel drug to reverse resistance to ADR is an important task in breast cancer chemotherapy [10].

Gambogenic acid (GNA), a dry gum-resin of the Garcinia genus, is a xanthonoid anticancer agent found in Gamboge [11]. It has been reported that GNA can inhibit cell proliferation by inducing apoptosis and cell cycle arrest by inactivation of the PTEN/PI3K/AKT signaling pathway in human tumors [12–15]. Mechanistically, GNA causes cell cycle arrest during the G0/G1 phase by inhibiting AKT phosphorylation and inducing the apoptosis of cancer cells via caspase-3. Thus, GNA could effectively inhibit the survival and proliferation of cancer cells [16]. Interestingly, the PTEN/PI3K/AKT signaling pathway was reportedly linked to chemotherapy resistance [17, 18]. For example, the experiment by Sokolosky [19] GSK-3β activity could result in the altered chemosensitivity of MCF-7 breast cancer cells to ADR through regulation of the PI3K/Akt/mTORC1 pathway by phosphorylating signaling molecules such as PTEN and TSC2.

Our previous studies have shown that GNA can induce apoptosis and inhibit proliferation in MCF-7 and MDA-MB-231 cell lines [20, 21]. In this study we provide preliminary evidence that GNA can increase the chemosensitivity to ADR in human breast cancer cells, at least in part, by inhibiting the Akt signaling pathway. Thus, GNA could serve as a modulator in treating ADR resistance in breast cancer patients.

## Methods

### Cells and cell culture

Human breast cancer MCF-7 and MCF-7/ADR cell lines were provided by Dr Jianwei Zhou (the Molecular Toxicology Laboratory, Nanjing Medical University) and cultured in Dulbecco’s minimum essential medium (DMEM, high-glucose) (Hyclone,Logan, USA) supplemented with 10 % calf serum (PAA, Ontario, Canada) at 37 °C with 5 % CO2.

### Reagents

Gambogenic acid (GNA) was purchased from Shanghai Ronghe Medical Technology Co. and was dissolved in DMSO (Sigma) to make a stock solution. The stock solution at 100 mg/ml was stored at 4 °C. MTT (3- (4,5-dimethylthiazol −2-yl)-2,5-diphenyltetra-zolium bromide) was purchased from Sigma Chemical Company (St. Louis, MO, USA). All other chemicals used were of the highest pure commercial grade available.

### Cell proliferation assay

Cell proliferation was determined using the MTT assay. The MCF-7 and MCF-7/ADR cells (5 × 10^4^) were seeded onto 96-well plates (Corning, Ithaca, USA). Four hours later, 10 μl of GNA in DMSO was added to the wells at various concentrations, and 0.1 % DMSO was used as a negative control. After 72 h, 50 μl of MTT was added, and the cells were incubated for another four hours. After the culture medium was removed, 150 ml of DMSO was added and the plates were placed on a shaking table at 150 rpm for 10 min. The optical density (OD) was measured at 490 nm. The experiments were repeated three times, and the rate of cell inhibition was calculated using the following formula: inhibition rate = [1-(OD test/OD negative control)] × 100 %. The IC50 was calculated using SPSS 19.0 software.

### Colony formation and clonogenic assay

The MCF-7 and MCF-7/ADR cells were seeded (1000 cells per well) in 6-well plates and grown at 37 °C in a 5 % CO2 incubator. Next, the cells were treated with ADR and/or GNA for 24 h, after which the drugs were washed out and fresh medium was added. After 2 weeks, colonies were fixed with methanol and stained with 0.1 % crystal violet (Sigma) in PBS for 15 min. Visible colonies were manually counted. Triplicate wells were measured in each treatment group.

### Cell cycle analysis

After treated with ADR alone or in combination with GNA for 48 h, cells were harvested, washed twice. The cells used for the cell-cycle analysis were stained with propidium oxide (100 μg/mL) using the Cycle Test Plus DNA Reagent Kit (BD Biosciences) and were analyzed by flow cytometry (FACScan; BD Biosciences) using an instrument equipped with the CellQuest software program (BD Biosciences). The percentages of cells in the G0–G1, S, and G2–M phases were counted and compared. All of the samples were assayed in triplicate.

### Apoptosis assay

Cells in the logarithmic growth phase were seeded onto 6-well plates to digest. The next day, pending adherent cells, seeded cells were added to the appropriate drug-containing medium accordingly, while the negative control group did not receive any durgs. After drugs administrations for 72 h, we collected cells via 0.25 % trypsin (without EDTA) digestion. The cells were washed twice with PBS (centrifuge 2000 rpm, 5 min), and we collected 5 × 10^5^ cells. We added 500 μL of a cell suspension in Binding Buffer, 5 μL of Annexin V-APC, and, finally, 5 μL of 7-AAD after mixing. At room temperature and protected from light, the mixture interacted for 5-15 min. Finally, we assayed for apoptosis using flow cytometry (Ex = 488 nm; Em = 530 nm).

### Western blotting analysis

Cells protein lysates were separated by 10 % SDS-polyacrylamide gel electrophoresis (SDS-PAGE), transferred to 0.22 μm NC membranes (Sigma) and incubated with specific antibodies. ECL chromogenic substrate was used to were quantify bands densitometry (Quantity One software; Bio-Rad). β-actin antibody (#3741, CST, USA) was used as a loading control, and anti-caspase-3(#9915, CST, USA), anti-caspase-9(#9502, CST, USA), anti-AKT(#9272, CST, USA), anti-p-AKT(#9275, CST, USA), and anti-PTEN(#9552, CST, USA) (all 1:1000) were purchased from Cell Signaling Technology, Inc (CST). The mean ± SD was calculated from three individual experiments. The gray scale of protein detection was analyzed using Gel-Pro32 software.

### Evaluation of combined effect and statistical analysis

The interaction between ADR and GNA was calculated and assessed using a combination index (CI): CI = D1/D×1 + D2/D×2. D1 and D2 are the concentrations of ADR and GNA that inhibited cell growth by × % when they were used in combination, respectively. DX1 and DX2 are the concentrations of ADR and GNA that resulted in a cell growth inhibition of × %, respectively. A CI < 1, CI = 1, or CI > 1 indicates synergistic, additive, or antagonistic effects, respectively. The data were analyzed using Calcusyn software (Biosoft, UK).

### Statistical evaluation

Values were expressed as the means ± standard deviations. Statistical analysis was performed using Student’s *t*-test. Values of *p* < 0.05 were considered to be statistically significant.

## Results

### Modulation of chemosensitivity to ADR in MCF-7/ADR Cells

To study the biologic mechanisms of chemosensitivity to ADR and find an opportunity to control resistance, we used an MTT assay to determine the IC50 values of ADR and GNA alone or in combination in MCF-7 and MCF-7/ADR cell lines. The results showed that ADR and GNA inhibited cell growth in a concentration- dependent manner (Fig. 1a, b). The combination of ADR and GNA enhanced the growth-inhibitory effect in MCF-7/ADR cells (cells were treated for 72 h), while the IC50 decreased from 4.31 μg/ml to 3.34 μg/ml (GNA1: 0.078125 μg/ml), 1.84 μg/ml (GNA2: 0.15625 μg/ml), and 1.45 μg/ml (GNA3: 0.3125 μg/ml) (Fig. 1d, e). Nevertheless, this phenomenon of an enhanced inhibitory ability was not observed in MCF-7 cells (Fig. 1c, e). This result indicates that the combination of ADR and GNA had a synergistic anti-tumor effect in MCF-7/ADR cells. The growth inhibition rates were analyzed using the Chou and Talalay method. The CI values were < 1, indicating that the combination of ADR and GNA had a synergistic growth-inhibitory effect in MCF-7/ADR cells (Fig. 1g). Similarly, this synergistic effect was not significant in MCF-7 cells (Fig. 1f).

**Fig. 1:** Growth inhibitory effect and combination index (CI) of ADR and/or GNA on MCF-7/ADR and parental MCF-7 cell lines. **a** Cellular inhibition rates were determined using the MTT assay. MCF-7/ADR cells were treated with various concentrations of ADR and GNA for 72 h. The group of MCF-7 cells was used as the control group. **b** Two cell lines were treated with ADR and various concentrations of GNA for 72 h. The cells treated with ADR alone were used as a control. **c** The IC50 values of two cell lines, which were treated with ADR and different concentrations of GNA, were measured using the MTT assay. According to the experimental results, the modulatory concentrations were as follows: GNA1:0.078125 μg/ml, GNA2:0.15625 μg/ml, and GNA3:0.3125 μg/ml. **d** The CI of the two drugs was determined using the Chou-Talalay method. CI < 1 indicates a synergistic effect. The data were presented as the means ± SD of three independent experiments. (** *P* < 0.01 and * *P* < 0.05)

### ADR and GNA alone and in combination inhibit MCF-7/ADR cell proliferation in vitro

The clonogenic assay was used to study the anti-proliferative effects of ADR and GNA in MCF-7 and MCF7/ADR cells. The results showed that ADR in combination with GNA significantly suppressed cell proliferation in MCF-7/ADR cells, but not in MCF-7 cells. As shown in Fig. 2, compared with the control cells, the combination of ADR and GNA in MCF-7/ADR cells resulted in markedly decreased colony formation abilities (*p* < 0.05). The colony formation of MCF-7/ADR cells was significantly inhibited from 107 to 43 and from 75 to 9, respectively, for 10 μg/ml ADR and 20 μg/ml ADR treatments alone or in combination with GNA.

**Fig. 2:** Effects of ADR and/or GNA on cell growth and proliferation of MCF-7/ADR (**b**) and parental MCF-7 cell lines (**a**). Colony-forming growth assays were performed to determine the proliferation of the two cell lines. The colonies were counted and captured. The data were presented as the means ± SD of three independent experiments. * *P* < 0.05

### The combination of ADR and GNA promotes G0/G1 arrest in MCF-7/ADR cell lines in vitro

To assess whether the anti-proliferative effects of ADR and GNA on the breast cancer cells were mediated by inhibiting cell cycle progression, we examined the cell cycling in MCF-7 and MCF-7/ADR cell lines by flow cytometry after treating the cells with different concentrations of ADR and GNA. The results demonstrated that the combination of ADR and GNA enhanced a significant arrest in the G0/G1-phase in MCF-7/ADR cells, with an obvious reduction in the number of cells in the S-phase, and this ability was not observed in MCF-7 cells (Fig. 3). In addition, these data indicate that ADR and GNA treatment could arrest MCF-7/ADR cells in the G0/G1-phase of the cell cycle with a concentration-dependent manner. Taken together, the combination of ADR and GNA exerts critical effects in MCF-7/ADR cell lines in vitro by affecting the cell cycle.

**Fig. 3:** Effects of ADR and GNA on the cell cycle of MCF-7/ADR and parental MCF-7 cell lines in vitro (* *P* < 0.05). **a** and **b** The bar chart represents the percentage of cells in the G0/G1, S, or G2/M phases, as indicated. The data represent the means ± S.D. from three independent experiments

### GNA increased the ADR-induced apoptotic rate in MCF-7/ADR cell lines

To further analyze how GNA affects ADR resistance, we assayed the apoptotic rates in two types of breast cancer cells by treating the cells with serial concentrations. The results showed that either ADR or GNA alone caused an increase in the percentage of apoptotic cells compared with the control group in MCF-7 and MCF-7/ADR cells. In the MCF-7 cell line, the apoptotic rates were increased from 76.3 % to 85.3 % (10 μg/ml ADR, 0.3125 μg/ml GNA) and from 80.3 % to 88.3 % (20 μg/ml ADR, 0.3125 μg/ml GNA). In the MCF-7/ADR cell line, the apoptotic rates were increased from 59.5 % to 71.1 % (10 μg/ml ADR, 0.3125 μg/ml GNA) and from 64.8 % to 75.1 % (20 μg/ml ADR, 0.3125 μg/ml GNA). By adding GNA, it was revealed that in MCF-7 and MCF-7/ADR cells, the number of apoptotic tumor cells was significantly increased in a dose-dependent manner, as determined using Annexin-V binding, strongly suggesting that GNA treatment caused an increase in apoptotic cell death by ADR (Fig. 4).

**Fig. 4:** The combined use of ADR and GNA significantly increased ADR-induced apoptosis in MCF-7/ADR cell lines (* *P* < 0.05). However, the proportion of increased apoptosis was not obvious in MCF-7 cell lines. The cells were exposed to different concentrations (0, 10, 20 μg/ml) of ADR with 0.3125 μg/ml GNA for 72 h. **a** and **b** The apoptotic rates of cells were detected by flow cytometry. Data represented the mean ± SD from three independent experiments

### Activation of ADR-induced apoptotic pathways induction by GNA

We next examined whether the GNA increased cytotoxicity of ADR was mediated by apoptosis. Our results showed that by adding 0.3125 μg/ml GNA and 20 μg/ml ADR to MCF-7/ADR cell lines for 72 h, the expression levels of the apoptosis-related proteins caspase-3 and caspase-9 were increased to varying degrees compared to the control group (Fig. 5). When GNA and ADR were combined at the concentrations indicated above, the expression levels of caspase-3 and caspase-9 were significantly increased compared to the ADR group, and the gray values were higher than the sum of the ADR and GNA groups. Thus, it was confirmed that GNA could activate the apoptosis-related proteins caspase-3 and caspase-9 to induce apoptosis in MCF-7/ADR cell lines, which modulated the resistance to ADR to some extent.

**Fig. 5:** MCF-7 and MCF-7/ADR cell lines treated with ADR + GNA showed up-regulated expression of caspase-3 and caspase-9. **a** and **b** Using either 0.3125 μg/ml GNA, 20 μg/ml ADR or the combined use of both ADR and GNA for 72 h, we used antibodies against caspase-3 and caspase-9 and analyzed the expression of caspase proteins by the western blot technique. β-actin was used as an internal control. (* *P* < 0.05)

### GNA altered the chemosensitivity to ADR via the AKT signaling pathway

To further clarify how GNA act as a regulatory factor to modulate drug resistance in MCF-7 and MCF-7/ADR cells, we adopted the western-blot method to investigate the Akt phosphorylation status and the expression changes in PTEN on the upstream PI3K/AKT pathway. As shown in Fig. 6, cells treated with GNA had enhanced expression of PTEN, a negative regulator of the PI3K/AKT pathway. Consequently, AKT phosphorylation was weakened without affecting the expression of total Akt. The expression of this protein downstream of the Akt signaling pathway was accordingly weakened, which might lead to the phenomenon of revering drug resistance.

**Fig. 6:** The application of ADR and GNA down-regulated the Akt signaling pathway in the MCF-7/ADR cell line. **a** and **b** Cells were treated with 20 μg/ml ADR, 0.3125 μg/ml GNA or 20 μg/ml ADR and 0.3125 μg/ml GNA for 72 h. Compared with the ADR group, the expression levels of p-AKT and PTEN in the ADR + GNA group were significantly increased to varying degrees (*P* < 0.05)

## Discussion

Breast cancer is a common type of cancer worldwide, and its incidence and mortality rates are rising, especially in premenopausal women [1–4]. ADR is the most effective anti-cancer agent commonly used in the clinic to treat various types of cancer, including breast cancer. With the wide application of ADR, the largest obstacle is its severe adverse side effects including multidrug resistance [22]. To eliminate this obstacle, we attempted to find a novel drug to reverse ADR resistance in breast cancer. In this study, two cell lines, MCF-7/ADR and its parental cell line MCF-7, were used to investigate the molecular biological mechanisms of chemotherapy resistance and also verified the regulatory function of GNA in MCF-7/ADR cells by MTT assay in vitro. We used an MTT assay to calculate the corresponding concentrations of the inhibitory rate after drug treatment. The results showed that the IC50 of a combination of GNA was significantly lower than that of the doxorubicin group alone and that the IC50 values declined with the increasing concentration of GNA in MCF-7/ADR resistant cell lines. Therefore, the effect of modulating the chemosensitivity of breast cancer cells to ADR was obtained.

Drug resistance is a major obstacle in chemotherapy. Resistant mechanisms in breast cancer are not entirely clear [23]. Research on the mechanism of resistance has been ongoing since the 1960s. In recent years, more thorough studies of the mechanism of drug resistance in breast cancer have shown that this process is very complex and requires multiple factors [24]. The PI3K/AKT pathway is an important signaling pathway that regulates cell proliferation, and AKT is a key molecule in the PI3K/AKT pathway [25]. When the extracellular signal near the cell membrane, receptor and ligand interactions lead to tyrosine kinase activation on the inner surface of the cell membrane. Further activation of phosphatidylinositol 3-kinase (PI3K) occurs, leading to mobilization at the cell membrane so that the substrate PIP2 (phosphatidylinositol4,5bisphosphate) can be converted to PIP3 (phosphatidylinositol3,4,5triphosphate). PIP3 is an important lipid second messenger required to phosphorylate AKT. Then, the phosphorylation of many proteins by P-AKT may be involved in the growth and development of cells [26]. PTEN is a protein phosphatase that acts on tyrosine residues, and is a major negative regulator of PIP3. Hypermutation of PTEN occurs in human tumors, including breast cancer, black melanoma, endometrial cancer and glioblastoma. PTEN has a dual phosphatase activity that regulates AKT and many downstream signaling proteins [27]. Inactivation of PTEN will lead to the activation of the PI3K/AKT pathway. Activation of AKT has many biological activities, such as, promotion of growth, proliferation, inhibition of apoptosis, enhanced invasion and metastasis, regulation of endothelial growth and angiogenesis through the catalysis of a series of protein phosphorylation events [28, 29].

Several studies have shown that GNA can inhibit proliferation through the induction of apoptosis in lung cancer cells [12, 30] and can induce mitochondria-dependent apoptosis in human hepatoma HepG2 cells [31]. Similar results from the A549 lung cancer cell line have been reported by Cheng H [13] and Yang L [14]. Our previous studies have shown that GNA can induce apoptosis and inhibit proliferation in the MCF-7 and MDA-MB-231 cell lines [20, 21]. To further explore the mechanism of GNA inhibition on proliferation in MCF-7 and MCF-7/ADR cell lines, we used flow cytometry to detect the cell cycle progression and apoptosis. The results demonstrated that a significant arrest in the G0/G1-phase and an obvious increase in apoptosis after adding GNA in MCF-7/ADR cells.

Clark’s [32] breast cancer research found that chemotherapy drugs can significantly activate PI3K, increase the levels of activated AKT, and cause cells to be antagonistic to chemotherapeutic drugs. Sokolosky’s experiment showed that inhibition of GSK-3β activity could result in altered chemosensitivity of MCF-7 breast cancer cells to ADR through regulation of PI3K/Akt/mTORC1 pathway activity by phosphorylating signal molecules such as PTEN and TSC2 [19]. These findings are consistent with other reports about the Akt signaling pathway in the role of breast carcinoma. These results strongly support the hypothesis that inhibition of excessive activation of Akt plays an important role in the reversal of chemotherapy resistance. In CNE-1 cells, gambogenic acid induced apoptosis through the inactivation of the Akt signaling pathway in human nasopharyngeal carcinoma [15]. Based on the experimental results above, we speculate that GNA reversed drug resistance by regulating the PTEN/PI3K/AKT signaling pathway, thereby affecting downstream target proteins. Here, we used the western-blot technique to detect three proteins involved in the PTEN/PI3K/AKT pathway as well as downstream proteins in MCF-7/ADR cell lines. We found that when combined with GNA in the MCF-7/ADR cell line, the expression of PTEN was significantly increased, the expression of phosphorylated AKT (i.e., excessive activation of AKT) was decreased, and the total AKT content did not change significantly. Then, we detected the expression levels of proteins affecting the cell cycle in MCF-7/ADR cell lines and found that they were significantly weakened according to gray-scale. Thus, GNA might act through the PTEN/PI3K/AKT pathways to inhibit resistant cell proliferation.

## Conclusions

This study demonstrated that GNA might inhibit the activation of Akt phosphorylation by acting on the negatively regulator of the AKT pathway, PTEN, to enhance its expression. Subsequently, apoptosis was induced in breast ADR-resistant cells, demonstrating that the chemosensitivity of breast cancer cells to ADR was modulated.
